The article "Learning to Discriminate Adversarial Examples by Sensitivity Inconsistency in IoHT Systems" was retracted in 2026. Reasons: signs of a paper mill; compromised peer review; suspected computer-generated content; unreliable results or conclusions.

# Learning to Discriminate Adversarial Examples by Sensitivity Inconsistency in IoHT Systems

**DOI:** 10.1155/2023/1177635

**Published:** 2023-02-22

**Authors:** Huan Zhang, Hao Tan, Bin Zhu, Le Wang, Muhammad Shafiq, Zhaoquan Gu

**Affiliations:** ^1^Cyberspace Institute of Advanced Technology, Guangzhou University, Guangzhou, China; ^2^Department of New Networks, Peng Cheng Laboratory, Shenzhen, China; ^3^School of Computer Science and Technology, Harbin Institute of Technology (Shenzhen), Shenzhen, China

## Abstract

Deep neural networks (DNNs) have been widely adopted in many fields, and they greatly promote the Internet of Health Things (IoHT) systems by mining health-related information. However, recent studies have shown the serious threat to DNN-based systems posed by adversarial attacks, which has raised widespread concerns. Attackers maliciously craft adversarial examples (AEs) and blend them into the normal examples (NEs) to fool the DNN models, which seriously affects the analysis results of the IoHT systems. Text data is a common form in such systems, such as the patients' medical records and prescriptions, and we study the security concerns of the DNNs for textural analysis. As identifying and correcting AEs in discrete textual representations is extremely challenging, the available detection techniques are still limited in performance and generalizability, especially in IoHT systems. In this paper, we propose an efficient and structure-free adversarial detection method, which detects AEs even in attack-unknown and model-agnostic circumstances. We reveal that sensitivity inconsistency prevails between AEs and NEs, leading them to react differently when important words in the text are perturbed. This discovery motivates us to design an adversarial detector based on adversarial features, which are extracted based on sensitivity inconsistency. Since the proposed detector is structure-free, it can be directly deployed in off-the-shelf applications without modifying the target models. Compared to the state-of-the-art detection methods, our proposed method improves adversarial detection performance, with an adversarial recall of up to 99.7% and an *F*1-score of up to 97.8%. In addition, extensive experiments have shown that our method achieves superior generalizability as it can be generalized across different attackers, models, and tasks.

## 1. Introduction

Recently, the fast development of deep neural networks (DNNs) has resulted in DNN-based models being applied in many scenarios around the Internet of Things, such as smart transportation [1, 2], intelligence healthcare [3], social networks [4], and information encryption [5, 6]. At the same time, the rapid proliferation of attacks against DNN-based models has raised greater security concerns [7]. Among them, adversarial attacks, which are novel and powerful, have caused harmful effects on model performance. In this paper, we study the security problems of the Internet of Health Things (IoHT) systems against adversarial attacks. As text data is a commonly adopted form in IoHT systems, such as the patients' basic information, medical records, and prescriptions, we focus on the security problems that may exist in such DNN-based textual analysis models.

The article "Learning to Discriminate Adversarial Examples by Sensitivity Inconsistency in IoHT Systems" was retracted in 2026. Reasons: signs of a paper mill; compromised peer review; suspected computer-generated content; unreliable results or conclusions.

As textual adversarial attacks exist in various forms and implement discrete perturbations, it has been a tough challenge to defend against such attacks in the DNN-based IoHT systems. Some defense methods against adversarial attacks have been proposed to address this challenge. The current approaches mainly focus on adversarial training [8, 9] and adversarial data augmentation [10, 11], which typically require retraining target models and extensive prior knowledge of attacks. Another type of defense method is input reconstruction [12, 13], which can be directly deployed into unmodified target models but hurts accuracy. In contrast, adversarial detection is a more direct defensive strategy that only detects adversarial examples (AEs) without correcting them [14–16]. In practical applications, this strategy has a high value because it alerts to threatening inputs and then rejects or submits them to other processing, rather than expecting the target model to give ambiguous and unreliable outputs. Obviously, adversarial detection is more appropriate in IoHT systems due to the hardware constraints. Unfortunately, very little attention has been paid to detection, and the available detection techniques are still limited in performance and generalizability.

In this work, we focus on adversarial detection. The goal of this study is to improve detection performance and generalizability. Based on sensitivity inconsistency to perturbation, we employ adversarial features, which are extracted from the shift of predicting labels and the similarity of probability distributions, to train a detector. The proposed method is efficient and high-transferable, which can catch AEs even in the circumstances of attack-unknown and model-agnostic.

We understand the difference between AEs and normal examples (NEs) in terms of geometric translation. An adversarial example can be regarded as a normal example changing along the adversarial direction. Geometrically, the adversarial direction usually points to the region where the decision boundary is highly curved [17]. Meanwhile, a study has pointed out that AEs easily lead to different classifications if fluctuations are caused at highly curved regions in the image domain [18]. Considering the goal of the attack, the adversarial examples are distributed centrally around the decision boundary to ensure low modification and imperceptibility. Thereby, we point to a common phenomenon: the AEs are boundary-sensitive. If we perturb the sensitive part of the AEs, it is extremely easy to cross the decision boundary. We consider important words (IWs) that contribute significantly to the decision as sensitive parts. As shown in Figure 1, if we intentionally perturb the IWs in examples, AEs easily lead to the target model making different predictions, while NEs maintain consistent behavior with the original.

The article "Learning to Discriminate Adversarial Examples by Sensitivity Inconsistency in IoHT Systems" was retracted in 2026. Reasons: signs of a paper mill; compromised peer review; suspected computer-generated content; unreliable results or conclusions.

To confirm this conjecture, we perturb the most important word in a set of AEs and NEs separately and illustrate the change in predictions of the model in Figure 2. As the result shows, in the NEs, perturbation of the most significant word leads to a shift in the probability values, but none crosses the decision boundary. However, in AEs, the same perturbation leads to prediction label changes in most examples. Further, the results show that even though the predicting labels of NEs change, the probability is closer to the decision threshold. It indicates that in NEs, the probability distributions in the Softmax layer are much closer before and after IWs are perturbed than those in AEs.

This preliminary work inspired us to design a detector trained with adversarial features that are extracted from perturbation-sensitive inconsistencies between NEs and AEs. We conclude that the sensitive inconsistency between NEs and AEs manifests in two parts: (1) whether the predicting label is changed after perturbing IWs; and (2) the inconsistency of the degree of change in probability distributions before and after perturbation. We combine the two points of sensitive inconsistency as the final adversarial feature. Our major contributions can be summarized as follows:

1. We propose an adversarial feature extraction method, named Sensitive Inconsistency Feature (SIF). As SIF is obtained from the universal differences between NEs and AEs, it can be generalized to different attack scenarios, even if they have never been known before.
2. We implement the adversarial detection method using SIF and machine learning mechanisms, named SIF Detector (SIFD). The experiments show our detection recall rate is up to a maximum of 99.7%, and the *F*1-score is 97.8% on IMDB, demonstrating its superiority over current advanced methods.
3. We present that SIFD exhibits transferability capabilities. In the most challenging settings (i.e., all of the configurations in the learning and detection phases are inconsistent), the *F*1-score and recall rates remain above 85%. All the codes to reproduce our experimental results are open source at https://github.com/AuroraHuan/SIFD-adversrial-detection and we hope they facilitate future research.

The article "Learning to Discriminate Adversarial Examples by Sensitivity Inconsistency in IoHT Systems" was retracted in 2026. Reasons: signs of a paper mill; compromised peer review; suspected computer-generated content; unreliable results or conclusions.

The remainder of this paper is organized as follows: Section 2 reviews the existing studies on adversarial attacks and defenses.  Section 3 describes the proposed detection method, SIFD. Experimental details, results, and analysis are given in Section 4. Finally, in-depth discussions and conclusions are given in Sections 5 and 6.

## 2. Related Work

This section briefly reviews adversarial attacks and defenses. As a hot research topic in recent years, there has been a lot of work on adversarial attacks. We focus on word-substitution attacks, which have received more attention as they perform better in semantic preservation and semantic correctness. Compared to other categories of attacks, word-substitution attacks better balance aggressiveness and concealability. As mentioned in the first section, we divide adversarial defenses into three categories, and in this section, we pay particular attention to adversarial detection, which is most relevant to our study.

### 2.1. Adversarial Attack

Given a text *x*, the attacker adds imperceptible perturbation *δ* to *x* to generate the adversarial example *x*_*adv*_=*x*+*δ* and aims to make the pre-trained model *F* misclassify, where the perturbation includes adding, deleting, and replacing characters or words.

#### 2.1.1. Gradient-Based Attack

As images are encoded as numerical vectors, perturbations generated by gradient sign methods are easily transformed into corresponding images [19–22]. However, these methods are not compatible with the textual domain because of the natural discreteness of texts. Therefore, for NLP tasks, gradient-based methods are usually combined with heuristic algorithms to generate adversarial examples, including the utilization of the value of the gradient to determine important words [23], sentences [24], or the ranking of perturbed substitutions [20, 25].

#### 2.1.2. Confidence-Based Attack

In this category, the attacker can obtain the classification confidence of each label. A common attack process includes two steps: (1) score the words according to confidence and sort them in descending order; and (2) sequentially perturb the sorted words until the attack succeeds or stops when it reaches the perturbation limit. The greedy search strategy is widely used to find optimal replacements in confidence-based attacks [10, 11, 26–28]. Besides, the genetic algorithm and bean search are also common search strategies [29, 30].

The article "Learning to Discriminate Adversarial Examples by Sensitivity Inconsistency in IoHT Systems" was retracted in 2026. Reasons: signs of a paper mill; compromised peer review; suspected computer-generated content; unreliable results or conclusions.

#### 2.1.3. Decision-Based Attack

The most challenging attack scenario is when the attackers only have access to the predicted labels of the target model. In this case, the attackers usually generate a weak adversarial example, followed by optimizing it until it generates a strong AE that is most similar to the original text [31, 32].

### 2.2. Adversarial Defense

#### 2.2.1. Robustness Enhancement

Gradient-based adversarial training is widely used for defense in the vision field [19, 21] with satisfactory effects, while in the natural language field it is effective in improving the accuracy and generalization of models [8, 33] but has weak gains in adversarial robustness. As a result, virtual adversarial training is widely used for textual adversarial robustness [9, 34, 35]. In addition, adversarial data augmentation [10, 27, 36] and virtual adversarial data augmentation [37] also effectively improve the adversarial robustness of models, but such methods are prone to decrease model accuracy. Zhu et al. [38] proposed a combination of friendly data augmentation and gradient-based adversarial training that can improve the adversarial robustness of models while maintaining their accuracy.

#### 2.2.2. Input Reconstruction

Discrete text is transformed into embedding vectors before input to the model, so many defense methods utilize reencoding to defend against spelling error attacks [36] and synonym attacks [39]. In addition, text-level reconstruction methods [12, 13] have been used to defend against word-substitution attacks. Among them, except for the method proposed in [13], the rest of the methods are effective for specific attacks and are not generalizable.

#### 2.2.3. Adversarial Detection

Different from the two types of defense methods mentioned above, adversarial detection only reports anomalies without correcting them. Although detections have been well used in the image domain [17, 40, 41], there are scarce studies on textual adversarial learning. Zhou et al. [14] trained a perturbation detector to detect potential perturbations and an embedding estimator to restore perturbations based on the BERT model [42], but trained by special AEs makes it difficult to generalize and the training of the BERT model is time-consuming. Mozes et al. [15] proposed detecting AEs through a simple and effective feature-word frequency, but this approach is only applicable to word-level attacks. Mosca et al. [16] trained a logit-based adversarial detector and achieved the best detection results in text classification so far.

## 3. Method

### 3.1. Overview of SIFD

Focusing on adversarial detection, the core of our idea is to extract distinguishable adversarial features and train a detector based on these features, and the overall process is shown in Figure 3. The intuition behind the approach is that even though AEs and NEs are extremely similar in semantics and visuals, they react inconsistently when important words are perturbed, i.e., the target model differs dramatically in output changes for AEs and NEs. The proposed method is divided into three steps: first, we inspect whether the predicting label has changed and mark it as a label inconsistency (*S*(*x*, *f*) in Figure 3); then we calculate the similarity of the probability distribution of the Softmax layer (*J*(*x*, *f*) in Figure 3); last, we combine features and train a detector.

The article "Learning to Discriminate Adversarial Examples by Sensitivity Inconsistency in IoHT Systems" was retracted in 2026. Reasons: signs of a paper mill; compromised peer review; suspected computer-generated content; unreliable results or conclusions.

### 3.2. The Feature of Sensitivity Inconsistency

For a given input text *x*=*w*_1_, *w*_2_,…, *w*_*n*_, including *n* words and the target model *F*, the process for extracting features is shown in Algorithm 1, including three main steps:

1. Ranking words and extracting IWs. We design an importance scoring function to rank the words in the text and select a specified number of IWs to participate in subsequent feature extraction.
2. Marking the word sensitivity signals. We define the concept of sensitive words for IWs and assign different values to sensitive and nonsensitive words.
3. Calculating the similarity of the probabilities distribution before and after perturbing IWs. Detailed explanations of the three steps are given in Subsection 3.2.1, 3.2.2, and 3.2.3, respectively.

#### 3.2.1. Ranking Word Importance

For attackers, regardless of the variations in the means of generating AEs, the ultimate goals are the same: minimizing the modification rate and maximizing the semantic similarity between AEs and their corresponding NEs, which are defined as the basic conditions of satisfying the adversarial example. To achieve these goals, attackers usually pick important words and perturb them, rather than make meaningless modifications to some unimportant words. Therefore, important words are powerful signals of the difference between the AEs and NEs, which consequently become the most critical features for adversarial detection.

Important words contribute much to the predicting of *F* so that the prediction probability changes significantly after removing it from *x*. We denote the contribution of a word *w*_*i*_ to *x* in model *F* by *I*(*w*_*i*_, *x*, *f*) which is usually expressed as

(1) $$\begin{array}{c} I\left(w_{i},x,f\right)=\left\{\begin{array}{ll} \left(x_{\backslash w_{i}},y_{i}\right)-f\left(x,y_{i}\right)+f\left(x,y\right)-f\left(x_{\backslash w_{i}},y\right)\text{,} & f\;if\;y_{i}\neq y\text{,}\\ f\left(x,y_{j}\right)-f\left(x_{\backslash w_{i}},y_{j}\right)\text{,} & others\text{,} \end{array}\right. \end{array}$$

where *x*_\*w*_*i*__ is text *x* that removes *w*_*i*_, *f*(*x*, *y*_*j*_) is the probability value of *x* to class *y*_*j*_, *y* is the predicting class of *x* according target model *F*, and *y*_*i*_ is the predicting class of *x*_\*w*_*i*__.

The article "Learning to Discriminate Adversarial Examples by Sensitivity Inconsistency in IoHT Systems" was retracted in 2026. Reasons: signs of a paper mill; compromised peer review; suspected computer-generated content; unreliable results or conclusions.

However, for a long text which consists of multiple sentences, this processing is time-consuming as it requires *n* forward calculation on *F*, where *n* is large. Our goal is to improve the efficiency of the processing. Following the study in [19, 23], we use the gradient magnitude to estimate the contribution of each word to prediction. The direction of gradient descent is the optimization signal to assist the model to obtain the minimum loss in the training phase; therefore, the word whose direction is close to the gradient contributes much to predicting *F*. According to this, we measure the importance of words by only 1 inquiry to *F*. Specifically, we utilize dot product to represent the angle between *w*_*i*_ and gradient on *w*_*i*_, which is calculated as

(2) $$\begin{array}{c} I\left(w_{i},x,f\right)=V_{w_{i}}∙\nabla_{w_{i}}J\left(\theta ,x,f\left(x\right)\right)\text{,} \end{array}$$

where *V*_*w*_*i*__ is the embedding of *w*_*i*_, *v* is the embedding dimension, and *J* is the loss function of *F*.

After ranking all words in *x* by equation (2), we further filter stop words from NLTK (https://ww.nltk.org/) and SpaCy (https://spcay.io/) libraries. Furthermore, we use NLTK to filter parts of speech, keeping only verbs, adverbs, adjectives, nouns, and their derived expressions, which correspond to the 16 lexical properties in NLTK. Finally, we select the most important *k* words as the feature source of text *x* for subsequent feature extraction, which is denoted as *C*(*x*).

#### 3.2.2. Marking Sensitivity Signals

AEs and NEs respond differently to the perturbing IWs. The predicting labels of AEs are highly susceptible to change due to the boundary sensitivity of AEs. In contrast, the probabilities for NEs in each class change, but the final predicting label remains relatively stable, which is similar to the principle of partial distortion of images without affecting the decision of the model [40]. Based on reaction inconsistency, we propose a method to define the sensitivity of the input *x*: for each word in *C*(*x*), we obtain the prediction classes before and after the word is removed, and then we define the word with different prediction classes as the sensitive word, and vice versa as a nonsensitive word. More precisely, the removal operation indicates the replacement of the original word as <MASK> for the pretrained models such as BERT and RoBERTa and <unk> for the traditional DNNs model such as LSTM and CNN. Furthermore, the set of signals based on sensitive words is adopted as the measure of the text sensitivity to *F*, denoted as *S*(*x*, *f*), which is formalized as

(3) $$\begin{array}{c} S\left(x,f\right)=\left\{s_{w}\left(x,x_{\backslash w_{i}},f\right)\right\}\;s.t.\;w_{i}\in C\left(x\right)\text{,} \end{array}$$

where *s*_*w*_(*x*, *x*_\*w*_*i*__, *f*) is a word-sensitive signal that is calculated as

(4) $$\begin{array}{c} s_{w}\left(x,x_{\backslash w_{i}},f\right)=\left\{\begin{array}{ll} 1\text{,} & if\;f\left(x\right)=f\left(x_{\backslash w_{i}}\right)\text{,}\\ -1\text{,} & if\;f\left(x\right)\neq f\left(x_{\backslash w_{i}}\right)\text{.} \end{array}\right. \end{array}$$

The article "Learning to Discriminate Adversarial Examples by Sensitivity Inconsistency in IoHT Systems" was retracted in 2026. Reasons: signs of a paper mill; compromised peer review; suspected computer-generated content; unreliable results or conclusions.

#### 3.2.3. Distribution Difference of Softmax Layer

It is not enough to rely on sensitivity signals alone to distinguish AEs and Nes, as discrete signals make it easy to cause many NEs to be incorrectly recalled as AEs. Furthermore, this error is more explicit in short-length texts because IWs in NEs are sensitive to perturbation. To solve this problem, we employ the inconsistency of the changes in probability distribution (i.e., the confidence scores of *x* predicted by *F* to all classes) of the Softmax layer as another feature. It signifies a more nuanced difference between AEs and NEs. Therefore, we use the Jensen-Shannon Divergence (JSD) to calculate this feature, which is expressed as

(5) $$\begin{array}{c} jsd\left(x,x_{\backslash w_{i}},f\right)=\frac{1}{2}KL\left(f_{s}\left(x\right)\|M\right)+\frac{1}{2}KL\left(f_{s}\left(x_{\backslash w_{i}}\right)\|M\right)\text{,} \end{array}$$

where *f*_*s*_(*x*) is the Softmax output, and *M* = (1/2)(*f*_*s*_(*x*) + *f*_*s*_(*x*_\*w*_*i*__) and *KL* is the Kullback–Leibler divergence, for which the formula is

(6) $$\begin{array}{c} KL\left(p\left\|q\right.\right)=\sum p\left(x\right)\log\frac{p\left(x\right)}{q\left(x\right)}\text{.} \end{array}$$

For each word in *C*(*x*), we calculate the JSD values according to equation (5) and use these values as the distribution variance features of *x*, denoted as

(7) $$\begin{array}{c} J\left(x,f\right)=\left\{jsd\left(x,x_{\backslash w_{i}},f\right)\right\}s.t.\;w_{i}\in C\left(x\right)\text{.} \end{array}$$

### 3.3. Training Detector

#### 3.3.1. Extracting of Distinguishable Features

The final input feature is calculated by combining the sensitivity flags *S*(*x*, *f*) and JSD values *J*(*x*, *f*)

(8) $$\begin{array}{c} E\left(x,f\right)=S\left(x,f\right)*J\left(x,f\right)\text{.} \end{array}$$

Thus, the input features for the adversarial detector are a set of continuum vectors of size *k*, and the labels are binary, 0 for NEs and 1 for AEs. In the training phase, we divide the data into a training set and a test set in the ratio of 8 : 2. In the test phase, the input features are computed by querying the target model *k*+1 times. Compared to the work in [16], which requires *n* queries, we save time costs in feature extraction and consider more distinguishable features. In Subsection 5.2, the advantages of combined features are demonstrated by ablation experiments.

The article "Learning to Discriminate Adversarial Examples by Sensitivity Inconsistency in IoHT Systems" was retracted in 2026. Reasons: signs of a paper mill; compromised peer review; suspected computer-generated content; unreliable results or conclusions.

#### 3.3.2. Design of the Detector

Following Mosca et al. [16], we do not fix detector architecture, and we train multiple machine learning models and evaluate their effects. Notably, our method does not depend on a specific model or a specific classification task, i.e., the detector can be deployed as a plug-and-play add-on to the target model to improve robustness. Moreover, although our detection method depends on the adversarial corpus, it is not limited to a specific attack method because the adversarial feature extraction method we design is based on the generic characteristics of AEs. Our proposed adversarial detection method is generalizable, which manifests in model agnostic, attack transportability, and data compatibility. In Subsection 4.4, we conduct an all-around analysis of the generalizability of our proposed method.

## 4. Experiments

### 4.1. Experiment Setup

#### 4.1.1. Datasets and Tasks

We adopt three popular classification benchmark datasets for our experiments: Internet movie reviews from IMDB [43], news articles on the web from AG's news [44], and the Yelp dataset challenge with polarity label [44]. As all of them are without a standard split for train/dev/test, we divide the original training set into training set and development set in a ratio of approximately 9 : 1. The statistics of them are shown in Table 1.

#### 4.1.2. Models

We adopt four DNN models that achieve state-of-the-art performance on text classification: BERT [42], RoBERTa [45], CNN [46], and LSTM [47]. Specifically, we use the pretrained BERT model and RoBERTa model with 12 transformer layers, 12 self-attention heads, and a hidden size of 768. We set dropout as 0.1 and epochs as 10, and fine-tune them with a batch size of 64 for AG's news and 32 for the others. The CNN model contains three convolutional layers with filter sizes of 3, 4, and 5. The LSTM model has 1 bidirectional layer and 128 hidden units. The inputs are initialized as embeddings by 300-dimensional pretrained word embeddings Glove [48] (https://github.com/stanfordnlp/GloVe) in LSTM and CNN. And the batch size is 256, the number of epochs is 20, and the dropout rate is 0.1 for both CNN and LSTM.

The article "Learning to Discriminate Adversarial Examples by Sensitivity Inconsistency in IoHT Systems" was retracted in 2026. Reasons: signs of a paper mill; compromised peer review; suspected computer-generated content; unreliable results or conclusions.

#### 4.1.3. Attack Methods

We employ four well-established attack methods: PWWS [26], TextFooler [10, 28], and BAE [27]. PWWS and TextFooler are the strong baselines for natural language attacks based on the black-box set and generate perturbation with synonym replacement; Deepwordbug crafts visual-similarity adversarial examples with a little number of typos; and BAE generates more semantic natural AEs by using the BERT masked language model. To ensure the consistency of attacks, we set the important parameters following the study in [8, 38]. The word modification rate is 0.2 for AG's news and 0.1 for the others, depending on the text length of the different datasets, and the threshold of the minimum similarity between AEs and NEs is 0.84 to ensure the reasonableness of AEs.

#### 4.1.4. Detection Baseline

We compare our proposed method SIFD with two other state-of-the-art detection methods FGWS [15] and WDR [16] under different combinational settings of datasets, models, and attacks. For FGWS, we follow all the detection settings of the original paper and determine the key parameter, threshold *γ*, which is the minimum value of the confidence difference for AE identification. For the IMDB dataset, we use the default threshold of 0.9 in the source code (https://github.com/maximilianmozes/fgws); for AG's news, referring to the tuning method and criteria in the original paper, we select *γ*=0.85 with the best true positive rate under the premise that no more than 10% of NEs are judged as AEs. Given that both our method and WRD are detector-based, we used a process similar to SIFD to train and test WRD. The architecture of the WRD detector is XGBoost [49], and the parameter settings are the same as those in the original paper.

#### 4.1.5. Evaluation Criteria

We employ several performance criteria to evaluate detection. We treat the AEs as positive examples (*P*) and the NEs as negative examples (*N*) for detection. Hence, *TP* denotes the number of *P* predicted as P, *FP* denotes the number of *N* predicted as P, *TN* denotes the number of *N* predicted as *N*, and *FN* denotes the number of *P* predicted as *N*. The criteria utilized in the experiment are as follows:

(9) $$\begin{array}{c} Recall=\frac{TP}{TP+FN}\text{,}\\ Accuracy=\frac{TP+TN}{TP+TN+FP+FN}\text{,}\\ F1-score=\frac{2*Precision*Recall}{Precision+Recall}\text{,}\\ Precision=\frac{TP}{TP+FP}\text{.} \end{array}$$

### 4.2. Detector Architecture Selection

We utilize multiple machine learning models as candidate architectures for the detector and compare their performances to select the model with the optimal detection performance for subsequent experiments. Specifically, we use BERT as the target model and fine-tune it on IMDB and AG's news, and then 1,500 adversarial examples generated by TextFooler for IMDB and PWWS for AG's news, separately. We extracted features from these AEs and their corresponding NEs, then divided the training, validation set, and test sets in proportions 8 : 1 : 1. Finally, we train and test five classifier models, including Random Forest [50], XGBoost [49], LightGBM [51], SVM [52], and AdaBoost [53].

The article "Learning to Discriminate Adversarial Examples by Sensitivity Inconsistency in IoHT Systems" was retracted in 2026. Reasons: signs of a paper mill; compromised peer review; suspected computer-generated content; unreliable results or conclusions.

As shown in Table 2, all the models achieve competitive detection performance, provided that all settings are identical. Among them, XGBoost performs slightly better, so we choose it as the detector architecture in the subsequent experiments. The main parameters of XGBoost include: the maximum depth is 3, the learning rate is 0.2, the gamma is 0.6, and other settings are disclosed in our open source code.

### 4.3. Detection Performance Comparison and Analysis

We compare SIFD with two advanced detection technologies. More specifically, we train and test the detectors in the same process as in Subsection 4.2, and for the nontrained FGWS, we test their performance in the tuned parameter settings. Although random sampling causes different examples to be selected each time, three detection methods compare their performance on the same examples in each configuration. As Deepwordbug is a character-level attack and FGWS detection is just designed for word-level attacks, we do not perform FGWS to detect adversarial examples generated by Deepwordbug.

As Table 3 presents, our proposed method outperforms the baseline method in 21 configurations (24 configurations in total). Even in the worse 3 configurations, the effect of our method is close to the optimal method. In addition, we observe that the effects of all detection methods on IMDB always outperform those on AG's news. To further clarify the causes of this phenomenon, we conduct a more detailed analysis in Subsection 5.3.

### 4.4. Transferability Evaluation

The transferability of the detector is a very important metric, as the data and models in the real-world defense phase are unpredictable and highly likely to be inconsistent with them in the training phase. In this subsection, unlike Subsections 4.2 and 4.3, we randomly sample 1000 texts (500 AEs and 500 NEs) to test the detection capability of the model for each configuration.

We first test the transferability of the detector on various attacks. Specifically, we first train the detector with the AEs generated by one attack and then test its ability to detect the AEs generated by other attacks. The detection effects with identical settings in the training and testing phases are seen as the baseline, which is called the default effect, and correspond to the row where the “^*∗*^” sign is located in Table 4.

The article "Learning to Discriminate Adversarial Examples by Sensitivity Inconsistency in IoHT Systems" was retracted in 2026. Reasons: signs of a paper mill; compromised peer review; suspected computer-generated content; unreliable results or conclusions.

As we can see from Table 4, our method always performs well in the migration from one attack to another. Both F1-score and adversarial recall rates differ from the default effect by a maximum of no more than 3%, and are always around ±1% and even sometimes better than the default effect.

Additionally, we test the transferability of different models. As shown in Table 5, LSTM and BERT exhibit remarkable transferability for each other, but the performance of CNN is relatively weak. We give a possible explanation for this phenomenon. We conjecture that the decision boundary of the trained CNN is more curved, and the convex region is steeper compared to the other two models. Therefore, the probability distributions vary greatly from AEs to their corresponding NEs. Therefore, the detectors learn features from these AEs that are significantly distinguishable and obtain excellent detection performance, but they struggle to detect more challenging AEs generated by other models. In addition, we observe that the attack success rate of various attack methods against the CNN model is higher than the others, and the adversarial recall ratio of detectors based on CNN is higher, which is consistent with our conjecture.

Furthermore, we consider the most challenging situation to be one in which all settings in the detection phase are different from those in the training phase. We select the detector trained by IMDB + BERT + TextFooler from Subsection 4.3 as the baseline detector and test it in two datasets, two models, and three attack methods. We trained the detector with IMDB + BERT + TextFooler and tested its detection performance with inconsistent datasets, models, and attack methods; the results are shown to the left of the parentheses in Table 6. As Table 6 shows, the scores for the two metrics are above 85% for various combinations of settings. It is worth noting that in some settings (bold in Table 6), the detection effect is better than the default effect (the values in parenthesis in Table 6), which needs further exploration.

## 5. Qualitative Results and Discussion

### 5.1. Impact of Important Words

We choose the most important *k* words to represent the input text for feature extraction. In this subsection, we study the effect of varying the value of *k* on the detection effect. As shown in Figure 4, for IMDB, recall and *F*1-score remain high at *k* ∈ [15,30], and then decline; for AG's news, scores reach the highest point at *k*=5. The results show that the best *k* values are different for texts and are tied to text length, and we suggest a range of [0.1*n*, 0.2*n*] and *n* is the length of text.

The article "Learning to Discriminate Adversarial Examples by Sensitivity Inconsistency in IoHT Systems" was retracted in 2026. Reasons: signs of a paper mill; compromised peer review; suspected computer-generated content; unreliable results or conclusions.

### 5.2. Impact of Features

We consider the effects of selecting top *k* IWs, sensitivity signal marking, and probability distribution differences on the final detection performance. We use TextFooler + BERT as the invariant setting of the experiment to test the detection effectiveness on AG's news and IMDB with different feature selections.  Table 7 shows the results of the ablation experiments, demonstrating that both the sensitivity signal and Softmax distribution inconsistency are effective as independent signals. Nevertheless, the best results are achieved by combining them. Individual sensitivity signs alone do not work well in short texts; by contrast, Jensen-Shannon divergence calculated by Softmax distribution differences plays a greater influence. In addition, the selection of top *k* IWs improves detection performance by 5 − 8%.

### 5.3. Impact of Datasets

Given the inconsistent capability of the detectors trained on IMDB and AG's news, we further explore exactly the key factor for this difference. The length of texts and the number of classes are two factors that are considered. In addition to the three datasets mentioned in Subsection 4.1, we add the SST-2 dataset as a reference experiment and split 5000 samples from the training set as the test set. Using four datasets and two baseline settings, we report the result in Table 8.

We observe a negligible difference in detection performance caused by the number of classes, but the data length matters detection performance a lot. We give a possible explanation for this phenomenon. In short-length texts with a small number of words, each word plays a more important role as texts have a small tolerance for information loss. As a result, perturbing each word in NEs affects higher fluctuations, so distinguishing between AEs and NEs becomes more challenging.

### 5.4. Challenges and Limitations

We propose the universal feature of AEs: sensitivity inconsistency to important words being perturbed. However, various still exist in examples reacting to perturbation across different datasets and tasks. We acknowledge that the detection effect is somewhat weakened in short-length texts. We argue that fuller features are beneficial to further improve the performance of the detector.

IWs play a big role in prediction, so attackers utilize them to craft AEs, which is a common pattern of attack. While SIFD contains rich information from IWs to identify AEs, its detection performance will be severely limited if a stronger attack method breaks this pattern in the future. Aiming to escape this cat-and-mouse game, our future work includes exploring certifiable defense methods with formal guarantees.

The article "Learning to Discriminate Adversarial Examples by Sensitivity Inconsistency in IoHT Systems" was retracted in 2026. Reasons: signs of a paper mill; compromised peer review; suspected computer-generated content; unreliable results or conclusions.

The proposed method, SIFD, can work not only as a detection plug-in to assist the target model but also in combination with others. Theoretically, the generality of SIFD motivates it to be combined with robustness training to jointly enhance adversarial robustness from inside and outside the model. In further research, we will explore more application potentials of detection against adversarial attacks.

## 6. Conclusions

We propose an adversarial detection method named SIFD based on sensitivity inconsistency features (SIF) against perturbing important words, which contain rich information for identifying AEs in DNN-based IoHT systems. Different from previous methods that identified features of detection from the whole text, we focused on only the important parts, which are the key features of texts, and achieved better distinguishable signals. The proposed method effectively enhances the adversarial robustness of the DNN-based IoHT systems in analyzing textual data.

We evaluate SIFD with advanced adversarial detection methods against four attack methods (both character-level and word-level attacks are included), and the results show the superiority of our approach over currently available detection technologies. In addition, through a series of ablation experiments, we reveal the remarkable transferability of SIFD and analyze the importance of each local mechanism in SIF.

## Figures and Tables

**Figure 1:** A visual illustrative example for sensitivity inconsistency of NEs and AEs against perturbing important words (IWs). The black arrow points to the direction of example movement (relative to the decision boundary) after IWs are perturbed. The figure shows that the perturbed AEs cross the decision boundary with high probability, but the NEs do not.

**Figure 2:** Visualization of probabilities values of NEs and AEs to the predicting label before perturbation. The AEs are generated by TextFooler attacking the CNN-based model. The *x*-axis and *y*-axis indicate the probability values for the true label before and after perturbation. Since the red line is *y*=0.5 and the IMDB dataset is a binary classification, the elements below the red line are examples that the predicting label changes.

**Figure 3:** The workflow of the proposed detection method SIFD.

**Figure 4:** Detector performance under different value of *k*, which is equivalent to the input dimension.

**Algorithm 1:** Feature extraction based on sensitivity inconsistency.

**Table 1:** Summary for datasets. #train, #dev, and #test count the number of texts in the train/dev/test set, respectively, #avg length is the average length of all the texts for each dataset, and #classes is the number of classes.

Dataset	#train	#dev	#test	#avg length	#classes	Task
IMDB	23,000	2,000	25,000	268	2	Sentiment analysis
AG's news	1,08,000	12,000	7,600	43	4	News classification
Yelp	5,00,000	60,000	38,000	152	2	Online reviews

The article "Learning to Discriminate Adversarial Examples by Sensitivity Inconsistency in IoHT Systems" was retracted in 2026. Reasons: signs of a paper mill; compromised peer review; suspected computer-generated content; unreliable results or conclusions.

**Table 2:** Detection performance of different machine learning model architectures. Bold values indicate the optimal results.

Dataset	Machine learning model	Accuracy (%)	Recall (%)	*F*1-score (%)
IMDB	Random forest	95.7	96.0	95.1
	XGBoost	96.1	**97.2**	**96.4**
	LightGBM	**96.3**	94.1	95.8
	SVM	92.3	93.2	92.1
	AdaBoost	95.2	96.0	94.9

AG's news	Random forest	89.5	88.1	89.0
	XGBoost	**92.7**	**91.9**	**92.2**
	LightGBM	91.7	80.4	91.3
	SVM	90.4	90.0	89.1
	AdaBoost	88.8	88.9	88.8

**Table 3:** Detection performance of three detection methods. The model, dataset, and attack method are consistent for the training and testing phases. As Deepwordbug is a character-level attack and FGWS detection is just designed for word-level attacks, the experimental results of Deepwordbug detection with FGWS are not meaningful, and “—” in the table indicates that the experiment is not conducted.

Model	Dataset	Attack	Recall (%)			*F*1-score (%)		
			FGWS	WDR	SIFD	FGWS	WDR	SIFD
BERT	AG's news	TextFooler	81.5	83.0	**91.7**	87.5	86.1	**90.7**
		PWWS	85.1	87.9	**91.9**	89.7	90.5	**92.2**
		BAE	49.7	80.0	**86.7**	57.2	81.2	**84.5**
		Deepwordbug	—	75.4	**85.0**	—	78.3	**85.6**
	IMDB	TextFooler	79.9	95.5	**97.2**	86.6	95.8	**96.4**
		PWWS	82.5	92.7	**95.5**	85.8	94.2	**96.0**
		BAE	56.7	90.3	**96.2**	67.8	93.1	**96.3**
		Deepwordbug	—	92.0	**94.2**	—	92.7	**94.8**

CNN	AG's news	TextFooler	82.9	92.0	**95.5**	86.2	89.7	**91.5**
		PWWS	86.8	91.0	**94.0**	91.2	86.0	**90.6**
		BAE	56.7	88.2	**92.4**	62.1	85.5	**88.5**
		Deepwordbug	—	91.0	**92.4**	—	**86.3**	84.9
	IMDB	TextFooler	75.9	89.9	**99.7**	85.3	91.5	**97.8**
		PWWS	80.2	87.2	**99.0**	86.0	87.2	**96.5**
		BAE	59.8	88.9	98.2	70.1	87.1	96.5
		Deepwordbug	—	91.2	**97.9**	—	89.6	**95.7**

LSTM	AG's news	TextFooler	86.2	91.3	**96.2**	90.1	87.8	**91.2**
		PWWS	84.7	84.6	**94.5**	90.4	86.8	**88.5**
		BAE	62.2	88.2	**91.7**	67.9	88.8	**90.3**
		Deepwordbug	—	83.4	**88.6**	—	83.3	**84.1**
	IMDB	TextFooler	77.4	94.8	**97.8**	83.8	95.0	**95.4**
		PWWS	70.5	**92.5**	92.0	80.0	92.4	**92.7**
		BAE	48.8	95.5	**96.9**	57.4	95.5	**97.7**
		Deepwordbug	—	92.0	**92.2**	—	**93.6**	91.5

Bold values indicate the optimal results among three defense methods.

**Table 4:** Generalization evaluation of different attacks. Rec is recall, *F*1 is *F*1-score, *R* is the variation of the current adversarial recall rate relative to the default effect, and *F* is the variation of the current weighted average *F*1-score relative to the default effect. ^*∗*^ denotes the baseline, which is the experimental setup for training the detector, followed by testing the detector against other attack methods with the same dataset and model.

Attack	CNN					LSTM				BERT			
	Rec (%)	&*R*(%)	*F*1 (%)	&*F*(%)	Rec (%)	&*R*(%)	*F*1 (%)	&*F*(%)	Rec (%)	&*R*(%)	*F*1 (%)	&*F*(%)
TextFooler^*∗*^	99.2	^*∗*^	96.3	^*∗*^	97.8	^*∗*^	95.4	^*∗*^	97	^*∗*^	97	^*∗*^
PWWS	98.2	+0.1	96.0	+0.8	91.7	−0.7	91.8	−0.4	95.4	−2.0	96.8	+0.3
BAE	99.2	+1	96.3	+0.5	96.5	−0.1	95.0	−0.8	93.2	−2.8	94.6	−0.9
Deepwordbug	97.4	−0.8	94.8	−0.4	92.0	0	91.8	+0.4	93.2	−3.0	94.9	−1.0

TextFooler	99.0	−0.2	95.5	−0.8	97.4	−0.4	95.8	+0.4	97.5	+0.5	96.2	−0.8
PWWS^*∗*^	98.1	^*∗*^	95.2	^*∗*^	92.4	^*∗*^	92.2	^*∗*^	97.4	^*∗*^	96.5	^*∗*^
BAE	98.8	+0.6	94.7	−1.1	97.2	+0.6	94.6	−1.2	95	−1.0	95.3	−0.2
Deepwordbug	97.8	−0.4	94.8	−0.4	92.2	+0.2	91.2	−0.2	94.6	−1.6	94.3	−1.6

TextFooler	98.8	−0.4	95.9	−0.4	96.9	−0.9	95.5	+0.1	97.4	+0.4	96.3	−0.7
PWWS	97.6	−0.6	96.4	+1.2	94.6	+2.4	93.9	+1.7	95.6	−1.8	95.7	−0.8
BAE^*∗*^	98.2	^*∗*^	95.8	^*∗*^	96.6	^*∗*^	95.8	^*∗*^	96	^*∗*^	95.5	^*∗*^
Deepwordbug	97.0	−1.2	94.7	−1.1	91.0	−1.0	91.9	+0.5	95.6	−0.6	95.3	−0.6

TextFooler	99.4	+0.2	96.3	0	95.8	−2.0	95.1	−0.3	97.8	+0.8	96.6	−0.4
PWWS	97.6	−0.6	95.6	+0.4	93.6	+1.2	91.7	−0.5	95.0	−2.4	95.7	−0.8
BAE	98.6	+0.4	95.3	−0.5	95.1	−1.5	94.3	−1.5	93.8	−2.2	93.9	−1.6
Deepwordbug	98.2	^*∗*^	95.2	^*∗*^	92.0	^*∗*^	91.4	^*∗*^	96.2	^*∗*^	95.9	^*∗*^

The article "Learning to Discriminate Adversarial Examples by Sensitivity Inconsistency in IoHT Systems" was retracted in 2026. Reasons: signs of a paper mill; compromised peer review; suspected computer-generated content; unreliable results or conclusions.

**Table 5:** Transferability evaluation of different models. Bold values indicate the better scores among two target models that model^*∗*^ migrate to.

Model	TextFooler		PWWS		BAE		Deepwordbug	
	Recall (%)	*F*1-score (%)	Recall (%)	*F*1-score (%)	Recall (%)	*F*1-score (%)	Recall (%)	*F*1-score (%)
CNN^*∗*^	99.2^*∗*^	96.3^*∗*^	98.1^*∗*^	95.2^*∗*^	98.2^*∗*^	95.8^*∗*^	98.6^*∗*^	95.5^*∗*^
LSTM	82.6	86.8	86.6	84.1	88.4	**90.9**	81.8	89.6
BERT	**89.2**	**93.8**	**91.6**	**92.6**	**90.4**	88.7	**89.7**	**92.5**

CNN	**98.5**	95.1	**99.9**	94.6	**97.5**	**94.8**	99.4	93.7
LSTM^*∗*^	97.5^*∗*^	95.4^*∗*^	92.1^*∗*^	92.2^*∗*^	96.5^*∗*^	95.5^*∗*^	92.3^*∗*^	91.6^*∗*^
BERT	97.2	**95.7**	95.0	**95.2**	91.8	93.3	**94.8**	**94.7**

CNN	**99.1**	**96.1**	**100.0**	**93.7**	**97.1**	**96.3**	**98.7**	**96.0**
LSTM	95.4	95.2	92.2	91.4	96.2	95.5	95.4	94.7
BERT^*∗*^	97.0^*∗*^	97.0^*∗*^	97.4^*∗*^	96.5^*∗*^	95.5^*∗*^	95.5^*∗*^	95.9^*∗*^	95.9^*∗*^

**Table 6:** Generalization evaluation in the toughest scenario. The values in parentheses are default effect. Bold values denotes that the detection performance under transferability is better than the default effect.

Dataset	Model	PWWS		BAE		Deepwordbug	
		Recall (%)	*F*1-score (%)	Recall (%)	*F*1-score (%)	Recall (%)	*F*1-score (%)
Yelp	LSTM	86.2 (91.6)	85.7 (90.5)	90.6 (94.5)	91.5 (93.2)	**92.8** (91.2)	**89.7** (87.4)
	RoBERTa	87.4 (94.7)	89.6 (92.6)	87.3 (92.0)	87.9 (92.7)	85.9 (92.8)	87.0 (89.1)

AG's news	LSTM	90.3 (94.4)	87.1 (88.5)	**93** (91.7)	**93.5** (90.3)	**91.4** (88.6)	**89.2** (84.1)
	RoBERTa	90.8 (91.3)	87.6 (85.4)	87.0 (89.9)	85.7 (91.2)	**88.9** (86.6)	**90.0** (87.5)

The article "Learning to Discriminate Adversarial Examples by Sensitivity Inconsistency in IoHT Systems" was retracted in 2026. Reasons: signs of a paper mill; compromised peer review; suspected computer-generated content; unreliable results or conclusions.

**Table 7:** Detection performance of different features. None means features dimensionality is 300 for IMDB and 100 for AG's news; in top *k* settings, *k*=20 for IMDB and *k*=5 for AG's news.

Top *k* IWs	Sensitivity flags	Softmax distribution	IMDB		AG's news	
			Recall (%)	*F*1-score (%)	Recall (%)	*F*1-score (%)
None	✓		80.0	89.5	78.6	72.3
		✓	92.4	94.1	84.9	87.6
	✓	✓	92.0	91.5	90.1	90.5

*k*	✓		84.4	92.4	76.9	77.5
		✓	95.2	96.1	89.4	90.7
	✓	✓	**99.8**	**97.7**	**95.5**	**91.5**

Bold values indicate the best results in different feature settings.

**Table 8:** Performance of detector on different datasets.

Dataset	BERT + Deepwordbug		LSTM + TextFooler	
	Recall (%)	*F*1-score (%)	Recall (%)	*F*1-score (%)
IMDB	94.2	94.8	97.2	96.4
AG's news	85.0	85.6	96.2	91.2
Yelp	90.1	92	95.5	93.4
SST-2	81.2	84.3	87.6	89.1

## Data Availability

All the codes and datasets to reproduce our experimental results are open source at https://github.com/AuroraHuan/SIFD-adversrial-detection, and we hope they facilitate future research.

## Additional Points

We confirm that this submission is not under consideration in any other journal, has not been published elsewhere, and is not currently under consideration by another journal.
